The article "Applications of Artificial Intelligence and Big Data Analytics in m-Health: A Healthcare System Perspective" was published in 2020. Journal: J Healthc Eng.

# Applications of Artificial Intelligence and Big Data Analytics in m-Health: A Healthcare System Perspective

**DOI:** 10.1155/2020/8894694

**Published:** 2020-08-30

**Authors:** Z. Faizal khan, Sultan Refa Alotaibi

**Affiliations:** College of Computing and Information Technology, Shaqra University, Shaqraa, Saudi Arabia

## Abstract

Mobile health (m-health) is the term of monitoring the health using mobile phones and patient monitoring devices etc. It has been often deemed as the substantial breakthrough in technology in this modern era. Recently, artificial intelligence (AI) and big data analytics have been applied within the m-health for providing an effective healthcare system. Various types of data such as electronic health records (EHRs), medical images, and complicated text which are diversified, poorly interpreted, and extensively unorganized have been used in the modern medical research. This is an important reason for the cause of various unorganized and unstructured datasets due to emergence of mobile applications along with the healthcare systems. In this paper, a systematic review is carried out on application of AI and the big data analytics to improve the m-health system. Various AI-based algorithms and frameworks of big data with respect to the source of data, techniques used, and the area of application are also discussed. This paper explores the applications of AI and big data analytics for providing insights to the users and enabling them to plan, using the resources especially for the specific challenges in m-health, and proposes a model based on the AI and big data analytics for m-health. Findings of this paper will guide the development of techniques using the combination of AI and the big data as source for handling m-health data more effectively.

## 1. Introduction

Mobile health is defined as the practice of applying mobile-based devices such as the mobile phones, patient monitoring devices, personal digital assistants (PDAs), and other wireless devices for the medical and public health. Therefore, this process requires the application of mobile phone's one of the most important benefits called the voice and short messaging service (SMS). At present, more than 500 projects are there for the m-health and nearly 40,000 medical-based mobile applications are also available worldwide [1]. There are mobile-based medical devices which are designed specifically for monitoring the heart rate [2], level of glucose [3], blood pressure [4], tracking the patterns of sleep [5], and also for monitoring the activity of brain [6]. It also uses more complicated operations and services such as the General Packet Radio Service (GPRS), 3rd and 4th generation mobile-based technologies, Global Positioning System (GPS), and Bluetooth-based technology. Big data [7–9] in the healthcare contains the medical images [10], clinical data of doctor, doctors' prescriptions and notes, computed tomography (CT) images, MRI scans, laboratory data, documents from the drugstore, files from the insurance EPR data, and other data related to the administrative operations. This is increasingly becoming favored within the worldwide communities of healthcare. However, there is a deficiency of understanding the most suitable framework based on the computational methodologies which are required for this approach. Big data analytics is the process of scrutinizing huge volume of data from various kinds of sources of data [11, 12]. These data are of different presentations and designs. Various analytical methods such as data mining and AI can be put in to examine the data. Approaches for big data analytics can be used to identify the abnormalities obtained as a result of combining large volume of data from different sources of data. Big data has become closely associative with the mobile health in recent years [13]. The main problems of big data analytics and the m-health are yet to be solved.

The article "Applications of Artificial Intelligence and Big Data Analytics in m-Health: A Healthcare System Perspective" was published in 2020. Journal: J Healthc Eng.

Various works have been done recently as proposals [14–28] or review [15, 27, 29–32] on m-health and applications of AI and big data analytics in healthcare sector. Applications of mobile phones have been successfully proven in medical-based applications for monitoring and have enhanced in the possibilities of assessing clinical data [27, 33]. Methods such as experience sampling methods (ESMs) and ecological momentary assessment (EMA) were applied in the process of assessing the patient's relationships between events and disease course [28]. These methods, which depend on providing contents which are informative in nature and questionnaires which were self-administered, reduce the recall since these applications will process in real time [34]. Recently, mobile devices can also able to perform passive gathering of data, i.e., to gather the information about the users without any effort on their part. Processes such as actigraphy, geolocation, and communication-based activities are usual features of current smartphones, and they can also be used in collecting the patient's behavior using the m-health-based systems. These m-health-based applications were also used to remotely monitor various physical and mental conditions [31]. Mobile-based health application can use various sensors for generating self-report of a patient. The authors in [26] proposed a mobile application for recognizing the human activity from inertial sensors to determine the user's activity level during the recording process. The signal from heart rate and galvanic skin response are also recorded in by their method to determine the emotional state of a user.

The article "Applications of Artificial Intelligence and Big Data Analytics in m-Health: A Healthcare System Perspective" was published in 2020. Journal: J Healthc Eng.

Following are the provocations that are still under consideration from the perspective of m-health:

- Better perception of the organized and unorganized sources of data produced from different sources of mobile and information.
- Smart implementation and conversion of the big data of health data occurred from the users of 5G mobile health. This should be performed in order to compare the most awaited intelligent and predefined change of behavior or convincing tools for inspiring more users for comfort and improvement of their health.
- Resilient, precise, and secure methods for data analytics for the explication of huge data of medical imaging and other relevant diagnostic data which are created and transferred from the future generation of mobile imaging devices should be developed.

The paper explores the applications of AI and big data analytics for providing insights to the users and enabling them to plan, uses resources especially for the specific challenges in m-health, and a proposes a model based on AI and big data analytics for m-health.

The remainder of the paper is organized as follows.  Section 2 shows the motivation and scope of this work along with the systematic reviews and meta-analysis process.  Section 3 depicts the definition of m-health and its schematic representation along with the mobile sensors and their applications in m-health.  Section 4 explains a detailed review about the applications of AI in m-health along with the performance measurement indicators used to examine the quality of m-healthcare.  Section 5 presents the applications of big data analytics in m-health followed by the additional summary of its applications in the healthcare sector.  Section 6 presents the proposed model based on the AI and big data analytics for m-health.  Section 7 depicts the limitations of the proposed review. Conclusion and the future enhancements are shown in Section 8.

## 2. Motivation and Scope

At present, there are many papers that have been published recently as proposals or review on m-health and applications of AI and big data analytics in healthcare sector. This paper outlines the characteristics and applications, scope/healthcare subarea, timeframe, and number of papers reviewed. This review is intended to answer the following research questions:

1. What is m-health and what sensors have been developed along with their applications for m-health?
2. What applications and benefits could AI technology bring to m-health?
3. What applications and benefits could big data analytics bring to m-health?
4. What are the challenges of adopting AI and big data analytics technology in m-health? anda proposed m-health model based on the combination of the AI and big data analytics.

The article "Applications of Artificial Intelligence and Big Data Analytics in m-Health: A Healthcare System Perspective" was published in 2020. Journal: J Healthc Eng.

The following sections describe how these questions were answered by this systematic review.

### 2.1. Methodology

The methodology of our review followed the checklist proposed by the Preferred Reporting Items for Systematic Reviews and Meta-Analyses (PRISMA) [35]. This review also identified applications of AI and big data analytics in m-health system. The review is limited to English articles and reports from 2007 to present date.

#### 2.1.1. Relevant Articles

Relevant articles and process of their selection for this systematic review are described in this section. In order to collect the relevant articles for this systematic review, we searched eight large scientific databases: the IEEE Xplore, ACM digital library, Taylor & Francis online, ScienceDirect, SAGE Journals, ProQuest, Springer, and Web of Science. This is done by an advance keyword searching process. The following terms were used in the search: “Artificial Intelligence AND m-Health,” “Big data analytics AND m-Health,” and “AI AND big data analytics in M-health.” Various articles were also found from the Google Scholar search. The main aim of this search is to find other quality articles that might be missed during the initial search in scientific databases.

#### 2.1.2. Inclusion and Exclusion of Articles

After completing the process of searching the article, the authors concealed the titles and abstracts of the retrieved articles using an inclusion and exclusion criteria. The articles that were not in English, the articles lacking full text, the articles that do not represent the applications of AI in m-health, the articles that do not represent the applications of big data analytics in m-health, and the articles with insufficient details were excluded. All the duplicate articles were removed. At last, 106 articles were obtained and kept for the review process. The above process is explained in the form of PRISMA flowchart in Figure 1.

### 2.2. Results

A total of 2543 articles were retrieved from the eight scientific databases. Then, another 130 additional articles were found through the search in Google Scholar. A total of 2437 articles have been excluded in the initial screening process. Among these, 1345 articles which do not represent the applications of AI in m-health, 902 articles which do not represent the applications of big data analytics in m-health, 78 articles which were from international journals, and 12 articles with insufficient details were excluded. Flowchart of the systematic reviews and meta-analyses (PRISMA) is shown in Figure 1.

The article "Applications of Artificial Intelligence and Big Data Analytics in m-Health: A Healthcare System Perspective" was published in 2020. Journal: J Healthc Eng.

## 3. Mobile Health

The application of mobile phones has inadequacies in infrastructure in developing countries which have led to huge changes in various healthcare sectors. Recently, mobile technology has played a significant role in various fields of technologies among various subscribers in almost all the countries. Mobile devices and communications assist the evolution of the proposed systems and their employment for the healthcare called m-health [36]. This comprises the combination of mobile devices, medical-based sensors [37], and portable devices [23, 38]. Health-based applications on smartphones are classified into the following: general health and fitness-based applications, information on medicine-based applications, and applications for managing the healthcare. m-Health is the innovative application of upcoming mobile-based technologies in concurrence with wearable devices especially in the application of healthcare informatics in order to enhance the practices of healthcare [39, 40]. m-Health has a scope of applying it to the mobile-based technologies. As a result, it produces various technologies such as the wearable devices, embedded systems, trackers for location, and legacy-based sensor devices. It also explores the facilitation in wireless-based communication [24, 41], ubiquitous computing, and other embedded technologies in healthcare to improve support of healthcare-based applications and also to reach into different pastoral areas [42, 43]. The schematic representation of m-health scenario is shown in Figure 2.

There are many advantages of using m-health. These devices can apprehend, save, recover, and transmit data to provide instantaneous, personalized informatics for individuals. m-Health could be a key element in healthcare systems [29] and can be useful in monitoring health status and improving patient safety and quality of care.

m-Health is becoming more popular in the smart device sector as it can provide remote assistance and data collection. Unlike an individual healthcare service, the collected data can be expanded and used across communities to understand common trends and thus improve the standards of healthcare. m-Health can provide support in vulnerable and remote communities via improvements to networks and the emergence of IoT [44].

The application of mobile technologies and their impact are likely to increase in the coming years. Surveys showed that mobile technologies and devices held about 80% of the overall global market in 2017, whereas in 2013, it was just 39%. The number of global users of smart mobile devices is anticipated to almost double in 2020 compared with 2014 and will reach 2.87 billion users [45]. This may increase the significance of m-health globally as shown in Figure 3. Low-cost smartphones have the required features and capabilities to cope with health-related applications and include the necessary connectivity [36].

The article "Applications of Artificial Intelligence and Big Data Analytics in m-Health: A Healthcare System Perspective" was published in 2020. Journal: J Healthc Eng.

As the popularity of m-health increases, countries are allotting more funding to this area helping society and communities to become more health literate. This promotes wellness rather than expensive medical intervention and hospitalization.

### 3.1. Mobile Sensors and Their Applications for m-Health

There are many mobile sensors which can be applied for a various applications of health [21, 47–52]. Various sensors such as camera sensor [53–55], microphone sensor [56–58], accelerometer sensor [59–61], and gyroscope sensor [59, 62] were used in the healthcare-based applications.  Table 1 shows a detailed outline of how the mobile-based sensors can be applied for various healthcare-based applications.

## 4. Applications of Artificial Intelligence in m-Health

Artificial intelligence is the process of demonstration of intelligence by machines in disparity to the natural intelligence depicted by the humans [24, 75, 76]. Machine learning is one of the applications of AI that lay out the systems to create capability to learn automatically and to enhance it from its training without being programmed explicitly. It also puts emphasis on the evolution of algorithms, can obtain data, and can adopt it for the process of making it to train themselves. Due to the fast enhancement of the AI, it has been employed in various fields, such as the IoT [22, 41, 77], machine vision [78], driver assistance [79, 80], and natural language processing [81, 82]. AI has been put in application in various domains of healthcare [83–87] which includes cancer research [88], cardiology [89], diabetes [90], mental health [91], identification of prognosis [92], identification of Alzheimer's disease [93], identification of difference in the clinical groups [94], identification of cardiovascular disease [39], stroke-related studies [95], etc.

Larburu et al. in [96] proposed an m-health application based on artificial intelligence for avoiding heart failures in patients. At present, the doctors are applying simple methods for generating alerts in the identification of heart failure. More false alerts are generated in the present methodology. In this work, predictive models were proposed to avoid the impact of these false alarms. These predictive models are based on clinical data taken from 242 heart failure patients' mobile accumulated in 44 months. The finest predictive model is acquired by the merger of various alerts which are based on observing the data and a set of questions using the application of a Naive Bayes classifier. This proposed model lowered the false alerts for a patient for a year from 28.64 to 7.8 gradually. In this method, the proposed system forecasts the possible risk of heart failures among the patients with more possibility of a heart failure. Main drawback of their method is that the accuracy of detection is less when the patient had undergone any heart surgeries in his past.

The article "Applications of Artificial Intelligence and Big Data Analytics in m-Health: A Healthcare System Perspective" was published in 2020. Journal: J Healthc Eng.

Burns et al. in [97] depicted the importance of mobile-based multicomponent that can be applied in the models of AI in order to analyze the different types of emotions such as the mood, cognitive state, depression, motivation, various activities, environmental behavior of the patient, and social behavior of the patient. Their proposed methodology gives graphs for feedback for the process of behavioral self-reflection, and it also provides coaching using various special trainers. The proposed methodology is based on the combination of regression along with decision trees and the phone sensor-based devices. Overall accuracy of their proposed methodology was excellent for the prediction of location about 60%–91%. Main drawback of their method is that the accuracy of prediction was very less for emotions, for example, sadness. In their analysis, they have selected eight patients for identifying the depressive disorder, the depression symptoms, anxiety, etc. Even though the accuracy of their proposed methodology is promising, the authors suggested the proposed methodology has to be enhanced since the outcome of prediction in the case of mood and location has to be upgraded.

Hawley et al. [98] proposed an application of automated machine in the recognition of speech of persons who are affected with dysarthria. It also assists in the process of voice message generation. In their method, the authors employed the hidden Markov models to decide the overall proximity of a word which is spoken to a speech model and is personalized for a particular person. Yet, the accuracy of their methodology for the speech recognition is only 67% for real-life study which comprises nine persons. The persons who participated identified that the hurdles in the process of communication are decreased by their proposed device when compared with the already available method of communication while speaking. Main drawback of their methodology is that its support is done by a usual aid for the voice-output communication and the accuracy of speech recognition hardware is less.

Martin et al. in [99] proposed a predicting and an alert generating methodology about multiple modalities such as lung diseases or cardiovascular problems in patients. Alerts were generated and sent to professionals of healthcare who can monitor the alerts based on the predefined guidelines. Their proposed system was based on the information collected through the phone calls of patients. Features such as linguistic and metalinguistic were extracted along with the status of patient in order to instruct the models of prediction. A 70% positive predictive value was obtained for unplanned events by their proposed methodology. Their proposed methodology was tested in a controlled manner with a set of 214 patients in a time period of six months. This is the biggest testing of an algorithm in terms of patient's participation and also with respect to the time taken. This methodology depicted a reduction rate of 50% in the number of participants in unplanned events of hospitals in the group when compared with custom alert generating mechanism.

The article "Applications of Artificial Intelligence and Big Data Analytics in m-Health: A Healthcare System Perspective" was published in 2020. Journal: J Healthc Eng.

Morrison et al. in [100] used the push notifications to upgrade the application of smartphone users for the process of stress management. The authors have employed a classifier called Naive Bayes for predicting the response of a user. Their algorithm predicts if a user would respond for a personalized intelligent mechanism for notification delivery when a notification is received from it. It depends on the number of times a user views and reacts within a day for the messages he received. This methodology was carried out for 72 hours which includes 76 participants. The drawback in this method is that the response is less when there is a distraction in the mobile networks.

Ortiz-Catalan et al in [101] used the pattern recognition algorithms for controlling the virtual limb movement in patients suffering from phantom limb pain. They also used gaming-based methodology combined with augmented reality for the process of treatment. Their proposed methodology was trained with a group of 14 participants. The results revealed that about 50% symptoms of phantom limb pain in patients were decreased significantly after 6 months of treatment. The authors also recommended that their novel method of treatment could be employed after clinical treatments. One of the disadvantages of their methodology is the time frame.  Table 2 depicts the additional summary of various applications of machine learning in the healthcare sector.

### 4.1. Performance Measurement Indicators Used to Examine the m-Healthcare Quality

In order to assess the quality of m-healthcare-based apps, various performance measurement indicators were proposed earlier. These performance measure indicators were proposed by incorporating the challenges of mobile health apps and strategies to ensure appropriate design and development of the apps for healthcare providers, patients, and the general public. Following are the various performance measurement indicators used to examine the quality of m-healthcare:

1. *Usefulness*. This metric enables the m-health user to achieve his or her specific goals and motivates the user to use the app repeatedly whenever necessary. This metric also analyzes how the mobile platform is effective in assessing how far the user is satisfied by the mobile healthcare system.
2. *Effectiveness*. Effectiveness is defined as the extent to which the m-healthcare system app works in the way that users expect it to and the ease with which users can apply it to achieve their specific goals. This is an important metric used in the case of m-healthcare quality.
3. *Veracity*. It is the measure of analyzing the accuracy and reliability of the information, data, or content present in the m-health application. Content in health apps is usually based on more than one source of information. The m-health application provides a method to enable the user to identify to the complete content more easily. Most of the m-health-based systems perform the functions of user or patient management, such as computation, tracking the data, and reminders, which should be more accurate.
4. *Interactivity*. It is the process of providing a sense of engagement with the user, entertainment, satisfaction to the patient or user, and motivation for the users who are using the m-health systems. It also extends to interactivity between service providers and patients as facilitated by the m-health app.
5. *Customization*. The main purpose of designing the m-health-based system is to support the users in one or more healthcare domains. Examples include assessment of diseases, its diagnostics, prevention of further complications, expert's intervention, and recovery. Customization is crucial in aiding the m-health-based system to achieve what the users intend to do. For example, the systems may have to connect to one or more EHR systems to provide the medical data of a particular user/patient.
6. *User Satisfaction*. User satisfaction can be defined as the proven willingness of a user for specified tasks in the overall m-health system or in using a specific system for repeated emergencies. This user acceptability has replaced most of the traditional metrics already available for assessing the usability in mobile health systems.

The article "Applications of Artificial Intelligence and Big Data Analytics in m-Health: A Healthcare System Perspective" was published in 2020. Journal: J Healthc Eng.

## 5. Applications of Big Data Analytics in m-Health

Recently, big data analytics has various options of providing advanced care for the patient and clinical decision support in the healthcare [14–17, 110, 111]. In general, application of big data in healthcare refers to the electronic datasets of health which are huge and complex and are difficult to manage with normal hardware, software, tools, and methods for managing the data [11]. Big data in the healthcare consists of clinical details of doctors, their notes and prescriptions, CT images, MRI images, laboratory data, documents from the drugstore, files from the insurance and other data related to the administrative operations, EPR data, etc. This comprises the big data. More methods have been proposed by various researchers to process these types of data. Still, there is a deficiency of understanding the most suitable framework based on the computational methodologies which are required for this approach. Hence, an enormous amount of data belonging to the healthcare is available for big data scientists. By understanding the advantages and disadvantages present in this, the big data analytics has to be enhanced in order to save the lives and to reduce the cost of processing data. Therefore, big data can be classified into two main categories [36] as follows:

- Organized data: in general, these data refer to the contents having defined format and length such as the numbers, generated date, and contents of strings. These data are formed by various sources such mobile phones, computers, various sensors, and logs of web. Examples of these types of data include EHR, home treatment and monitoring data, prescriptions from the doctors, etc.
- Unorganized data: in general, these data refer to the contents which do not have a predefined format of big data. The majority of the data are generated from various sources, such as the data from social media, mobile data, and content from the video and web. Examples of unorganized health data include health data from the social platform such as from Twitter, Facebook, user blogs, notes of clinicians, and diaries of medication and its instructions.

The process of analyzing a huge amount of data from various sources of data and different formats in order to convey the perception of enabling a decision-making process in real time is called big data analytics. Various concepts of analytics such as data mining and AI can be used to analyze the obtained data. These analytical approaches in big data can be used to identify the anomalies by analyzing a huge amount of data from various datasets and their sources.  Figure 4 shows an example of the smartphone-based m-health model with the combination of AI and big data analytics. Nowadays, the conversion of digital version of all exams done in clinical and medical fields yields huge data and records, which has formed a standard and has been widely accepted and implemented in practice.

The article "Applications of Artificial Intelligence and Big Data Analytics in m-Health: A Healthcare System Perspective" was published in 2020. Journal: J Healthc Eng.

EHRs are defined as the computerized form of medical records for all the patients. It has various information regarding the previous, current, and upcoming physical and the mental health situation of an individual. These electronic systems are used to apprehend, transfer, obtain, stock, connect, and change the data of multimedia. The primary purpose of this electronic system is to provide services related to the health [45]. Main advantages of these EHRs are that they enable faster retrieval of data and the professionals in healthcare have an enhanced access to the whole history of the patient about his medical details. Its benefits include providing better healthcare by making better classifications of the patient's health.

Similar to EHR, another record called electronic medical record (EMR) is used to store the medical and clinical data which are gathered from the patients. These are standard in nature. EHRs, EMRs, PHR, software for the medical practice management, and various other components of the healthcare data increase the quality and efficiency of service and reduce the overall cost of healthcare and medical errors. The healthcare big data consist of the data from healthcare provider and various experiments done in the laboratories and various other data obtained from the IoT-based devices.

Raghupathi and Raghupathi [112] proposed a novel architecture for the healthcare-based system applying the analytics of big data. Their methodology comprises various layers for data source, transformation, big data platform, and analytics. The layer for data source mainly focuses on the data sources of internal and external healthcare which can be found in different locations and in different formats. The layer for transformation is accountable for various tasks such as removal, conversion, and uploading of data in the platform of big data for the process of doing specific operations on the Distributed File System using a programming model called Map-Reduce. The main task of analytical layer is to do various operations such as inquiring, announcing, online analytical processing, and mining the data.

A patient-centric personalized framework for healthcare based on the collaborative filtering approach was proposed by Chawla and Davis in [113]. It apprehends the similarities in different patients and generates the personalized profiles for risky diseases for individuals. Collaborative filtering is one form of data analysis technique which is designed to guess the opinion of user regarding an entity item or its service; it is based on the preferences from a known group of a large number of users. In their framework, healthcare history of individual patients was collated with all the medical histories of other available patients. This is based on the following similarity constraints. Some of these are occupation, symptom, result from the laboratory, history of family, data of demography, etc. Based on the computation of similarity, a collection of patients who are similar is chosen and the prediction of diseases is done. Since the application of electronic healthcare records was increased, their framework depicts a proactive healthcare solution with respect to the context of big data. Even though their proposed methodology has various advantages, their proposed methodology handles only the identification of codes for various diseases.

The article "Applications of Artificial Intelligence and Big Data Analytics in m-Health: A Healthcare System Perspective" was published in 2020. Journal: J Healthc Eng.

An analytical framework of big data that employs ubiquitous healthcare system was proposed by Kim et al. in [114]. Their proposed framework analyzes the vital signs obtained from accelerometers in order to provide healthcare services. Vital signs are continuous time series data which are unstructured in nature having inadequacy to be stored in the traditional databases. Data obtained from ECG and from the respiratory system are considered as vital signs. Their proposed framework used a platform of open standard in order to support the inability of data exchange between various devices. This platform has been enlarged by including various algorithms for the process of extracting feature values from the fresh vital signs data and then storing them for the process of real-time analysis. Even though their proposed methodology has various advantages, their work has a major disadvantage in delivering considerable analytical models.

A detailed survey on the inference of computational methods in the big data-based health informatics has been done by Fang et al. in [30]. They focused on a novel framework called “Health informatics processing pipeline” which incorporates various steps to obtain significant patterns from healthcare-based big data. Their proposed framework consists of pipeline process such as capturing the data, storing the data, analysis, extraction, and decision support systems. Apart from the proposed framework, some directions for research in the heterogeneity of data such as organized and unorganized data of the healthcare, existing complexities which are available in the available data, issues of privacy, and analysis of the identified patterns are also traversed in their entire work. Their proposed healthcare-based framework offers a systematic pipeline of data processing for various stages of informatics of big data such as data acquisition, saving, finding, and analyzing data from diversified sources. Hence, the authors focused on enhancing the aspects of technological development by using the tools and techniques of big data. Due to the enhancement of mobile devices and wireless sensor networks, healthcare services were improved. As a result, the services are offered at any time and at anywhere in the health informatics domain.

The article "Applications of Artificial Intelligence and Big Data Analytics in m-Health: A Healthcare System Perspective" was published in 2020. Journal: J Healthc Eng.

Pramanik et al. in [115] performed a detailed analysis on the latest improvements in healthcare-based systems. Their work mainly focuses on the applications of technologies based on smart system. They focused on a novel framework for the smart healthcare system enabled by big data for maintaining ubiquitous solutions for healthcare. It also offered a reduced cost with improved advancements. It consisted of the following layers:

- Data source layer: designed especially for maintaining the organized, unorganized, and semiorganized data sources.
- Data analytics layer: designed mainly for processing calculations on big data, its visualization, and management.
- Smart service layer: designed mainly for making ease of various favors such as the monitoring of data, agreement on privacy, and security between the providers, consumers, and their services. Also, this layer proposes various smart services and their infrastructure with the help of various devices and software.
- Knowledge discovery layer: improved functionalities such as the guessing necessity of entities, proposal, and its cost evaluation of mechanism for providing the healthcare service were also included.

The authors proposed a framework for the organizations in healthcare in providing intelligence-based smart services. Their detailed research depicts a novel framework for the smart healthcare system based on big data and also makes the research directions interdisciplinary. In fact, the proposed framework is the combination of three technical streams such as the AI, agent-based systems, and data mining along with the smart health. Additional summary of the applications of big data in the healthcare sector is provided in Table 3.

## 6. Proposed Model Based on AI and Big Data Analytics for m-Health

The proposed framework comprises three essential parts such as the medical data obtained from the patients through the mobile phone and the telemonitoring devices, AI and big data analytics platform, and the output towards the mobile care monitor. The architecture of the proposed system is shown in Figure 5. The entire process of analyzing a huge amount of data obtained from various sources of data in different formats is processed by the combination of AI and big data platform. These are combined to convey the perception of enabling a decision-making process in real time. Various concepts of analytics such as data mining and AI are used to analyze the obtained data from a patient. These analytical approaches in big data can be used to identify the anomalies by analyzing a huge amount of data from various datasets and their sources such as biomedical signals, physiological sensing data, genomic data, and biomedical imaging. The AI-based engine comprises two modules such as the stream analysis module and the AI-based report management tool. These analyze the queries obtained from the big data analysis engine.

The article "Applications of Artificial Intelligence and Big Data Analytics in m-Health: A Healthcare System Perspective" was published in 2020. Journal: J Healthc Eng.

The main aim of the AI-based report management tool is to generate a better decision using the AI technology in order to report the status of the patient's health. It is also used as a platform for the disease control, treatment, and diagnosis tool. In this model, the AI-based report management tool collects, analyzes, performs, and triggers the action by classifying the code of a disease or condition using the free text approach. It also extracts the features from the EHR. It also detects the irregular records which are present in the EHR. All the processed streams are stored and updated in the big data engine.

The big data analysis engine consists of two modules such as storage for big data and a statistical data analysis tool. The statistical data analysis tool retrieves the input data, processes it into queries, and then sends it to the AI-based engine. All the processed queries and streams were given as output towards the mobile care monitor.

The proposed model enhances the overall performance of m-health since AI and big data analytics are combined. The proposed methodology improves the process of m-health by processing each and every query, and it also enables a decision-making process in real time.

## 7. Limitations

Despite the various advantages of the proposed m-health model based on AI and big data analytics, some limitations were also there that need to be considered: a large section of population, system can never be too accurate, have to depend completely on the technology, and several privacy and security issues.

With regard to a large section of population, the access to m-health-based system is denied because of their numbers, their incapacity to afford it, and the lack of knowledge and skill to use it. The system can never be too accurate to replace the humans and their predictions. These systems have been made to ease out the health structure but they cannot be a substitute to human. Even the most well designed and technologically best developed apps can also never be hundred percent accurate.

These m-health systems also make a user/patient to be dependent completely on them. If the user loses his or her mobile phone and user id/password, there is a possibility for all the information to be lost temporarily or even permanently. There might be a chance for various issues in the privacy and security of the health data present in it. In such cases, there is a chance for the personal information to be leaked and shared to unauthorized users.

The article "Applications of Artificial Intelligence and Big Data Analytics in m-Health: A Healthcare System Perspective" was published in 2020. Journal: J Healthc Eng.

## 8. Conclusion and Future Works

m-Health is a technique which uses mobile devices and technology for health interventions and is the biggest technological advancement of recent research. Similarly, the application of AI and the analytics of big data in healthcare are considered as one of the important achievements for the intelligent healthcare system. In this paper, a detailed review of the m-healthcare system is proposed based on the application of AI and big data analytics. Various advantages from this combination for the m-health perspective are presented. Particularly, all applications of relevant technological areas and the building blocks such as communications, sensors, and computing which are associated with mobile health are explained in detail. The role of various tools of machine learning within the current m-health model is also illustrated. Future works can be a comprehensive review on the retrospective validation of models of the AI and combining them with various digital health tools and evaluating their clinical validation and efficacy issues on these systems. Future works can be the proposal of application of intelligent agent-based systems for providing privacy and security in m-health big data.

## Figures and Tables

**Figure 1:** PRISMA flowchart for the entire review process.

**Figure 2:** Schematic representation of the m-health scenario.

**Figure 3:** Global m-health markets [46].

**Figure 4:** Smartphone-based m-health model with AI and big data analytics.

**Figure 5:** Architecture of the proposed AI and big data analytics-based m-health system.

**Table 1:** Mobile-based sensors applied for various healthcare-based applications.

Mobile sensors	Main area	Applications in healthcare
Camera	Capturing photo and video	Applied for identifying various categories of diseases, in the perspective of effects in surgery, diagnosis of diseases, observing the slash, analysis of skin disease [63], monitoring the health of child, etc. [18].

GPS	Location tracking	Provides an access to follow the patients who are vulnerable to some diseases such as the people with Alzheimer's disease [64] and Ebola [65] by the application of mobile-based applications [66].

Electrocardiograph	Cardiovascular disease monitoring	Mobile phones which are enabled with the electrocardiographs are being used in areas which are underdeveloped for the purpose of monitoring the patients with heart diseases [40, 67].

Bluetooth	Data sharing and communication	It allows a midrange data communication between mobile devises, various other healthcare monitoring devices, and wearable sensors.

Microphone	Voice recording	It allows the doctors to communicate with the patients regarding the support for identification and treatment of diseases. It also comes up with the way for analyzing the audio for assessing the feeling of a patient with various diseases such as muscular dystrophy [68].

Accelerometer	Acceleration measurement	It assists to compute the orientation of devices which are relative to Earth especially for calculating the motion. It can be executed in various activity monitoring techniques of patients such as counting the step of a person, gait analysis, and monitoring [19, 69].

Wi-Fi	Data sharing and communication	Wi-Fi-based mobile sensor enables the mobile device to communicate with the physician about the healthcare data to for the purpose of identification of a disease and its treatments.

Accelerometer, GPS, compass, gyroscope, and barometer	Physical activities	Combination of hardware and the sensors present in it is being utilized for computing the stationary vs nonstationary actions [20].

Microphone, accelerometer, and GPS	Social engagement	This combination makes the monitoring of psychological health by checking the social problems, talks from the conversationalists, consternation, strain, behaviors related to depression, etc. [70, 71].

Microphone, GPS, accelerometer, touch interface, and light sensor	Sleep pattern tracking	Combination of this hardware depicts the data of interrupted vs constant patterns of sleep in a patient [71–74].

The article "Applications of Artificial Intelligence and Big Data Analytics in m-Health: A Healthcare System Perspective" was published in 2020. Journal: J Healthc Eng.

**Table 2:** Additional summary of the AI methods suitable for the healthcare sector.

Name of the framework	System	Technique	Area of application
Apache Mahout [102]	Library for machine learning (open source)	A real-time computation system which is more flexible and scalable.	Provides mechanisms such as clustering, classification, and regression.

Skytree [103]	AI-based platform which is applied for general purpose algorithms	Applies artificial intelligence for producing complicated algorithms for more advanced analytics.	For processing very large organized and unorganized datasets more accurately without performing downsampling.

Karmasphere [104]	Platform of big data	Searches and scrutinizes the web-based, mobile-based, and sensor-based data in Hadoop for the social media.	Develops and issues a graphical-based environment which assists the way finding through any type of big data and identifies the recent trends and patterns present in it.

BigML [105]	Platform for AI-based programs	Gives various tools for performing tasks related to AI such as clustering, regression analysis, pattern classification, detection of anomaly, and discovery of association.	It combines the AI-based features along with the cloud-based infrastructure for developing applications which are cost-effective, highly accurate, reliable, and flexible.

Cognitive machine learning algorithm [106]	Cognitive computing tool	Associative memory classifier-based machine learning algorithm.	Echocardiography data are normalized using the machine learning algorithm in order to differentiate the constrictive pericarditis from restrictive cardiomyopathy.

Machine learning algorithms [107]	Support vector machine	Analyzes and classifies a multidimensional echocardiographic data based on gap in present in it.	To distinguish between athlete heart and hypertrophic cardiomyopathy.

Phenotypic clustering [108]	Hierarchical clustering	Classifies similar objects between the same clusters and calculates the hierarchy in the echocardiographic data.	To analyze the clustering of echocardiographic variables in order to compute the dysfunction in left ventricular and isolate high-risk phenotyping patterns.

Convolutional neural network [109]	Combination of AI and natural language processing	It reads the chest X-ray reports of patients and assists the antibiotic assistant system to alert physicians for anti-infective therapy.	It combines the AI-based features along with the natural language processing for effective diagnosis of diseases.

**Table 3:** Additional summary of the applications of big data in the healthcare sector.

Name of the framework	Source of data	Technique	Area of application
Substructure for preserving privacy in healthcare systems based on RFID [116]	Data produced from the tags of RFID	Privacy preservation methods	Reliable healthcare-based services. Enhanced isolation in healthcare system based on RFID.

Novel framework for distributed and secured HIS [46]	Electronic-based health records	Providing security limitation and control mechanisms for accessing the data	Secure healthcare system. Distributed and secured multitier framework.

Smart framework for healthcare system enabled with big data [115]	EHR, report on diagnosis, data from the social media, biometric data, and monitoring data	Providing services of smart healthcare by infrastructure which is service oriented	Technologies based on smart system especially for the healthcare system. Combining the healthcare knowledge data mining strategies with the infrastructure of smart services.

Framework for policy enforcement towards IoT-based smart health [117]	Patients' various biological parameters, data related to environmental factors, and data generated from the instruments such as RFID	Providing access control based on policy mechanism for offering resources of healthcare	Smart health applications for avoiding threats in security for large scale and heterogeneous scenarios.

Framework for prediction of protein structure using big data and ensemble learning [118]	Protein structure dataset	Ensemble learning technique based on distributed tree	Design of drugs. Depicts a distributed framework with enhanced accuracy.

Framework for smart health [44]	Datasets of the patient from various sources such as the health information system and the radiology department	Pattern recognition and its matching techniques	Big data-based analytics for the applications of smart healthcare. Improving the services of healthcare by combining the sensor-based technologies along with the cloud computing and big data analytics.

A semantic web-based technology for maintaining and reusing the archetypes present in clinical data [119]	EHR	Building the ontology through ontology web language	Classification of patient based on various clinical criteria. Combining the semantic-based resources along with the EHR.

The article "Applications of Artificial Intelligence and Big Data Analytics in m-Health: A Healthcare System Perspective" was published in 2020. Journal: J Healthc Eng.

## Data Availability

The data that support the findings of this study are available from the corresponding author on request.
